RETRACTED

# SSRP1 promotes colorectal cancer progression and is negatively regulated by miR‐28‐5p

**DOI:** 10.1111/jcmm.14134

**Published:** 2019-02-14

**Authors:** Wei Wu, Ke He, Qian Guo, Jingdi Chen, Mengjiao Zhang, Kai Huang, Dongmei Yang, Lu Wu, Yunchao Deng, Xu Luo, Honggang Yu, Qianshan Ding, Guoan Xiang

**Affiliations:** ^1^ Department of Critical Care Medicine Renmin Hospital of Wuhan University Wuhan Hubei P.R. China; ^2^ Department of Gastroenterology Renmin Hospital of Wuhan University Wuhan Hubei P.R. China; ^3^ Hubei Key laboratory of Digestive System Renmin Hospital of Wuhan University Wuhan Hubei P.R. China; ^4^ Department of General Surgery The Second People's Hospital of Guangdong Province, Southern Medical University Guangzhou Guangdong P.R.China; ^5^ Hepatic Disease Institute, Hubei Provincial Hospital of Traditional Chinese Medicine Wuhan Hubei P.R. China; ^6^ Department of orthopedics The Airborne Military Hospital Wuhan Hubei P.R. China; ^7^ Eppley Institute for Research in Cancer and Allied Diseases Fred and Pamela Buffett Cancer Center University of Nebraska Medical Center Omaha Nebraska; ^8^ School of Electrical and Electronic Engineering Nanyang Technological University Singapore

**Keywords:** colorectal cancer, microRNA, progression, SSRP1

## Abstract

In this study, microarray data analysis, real‐time quantitative PCR and immunohistochemistry were used to detect the expression levels of SSRP1 in colorectal cancer (CRC) tissue and in corresponding normal tissue. The association between structure‐specific recognition protein 1 (SSRP1) expression and patient prognosis was examined by Kaplan‐Meier analysis. SSRP1 was knocked down and overexpressed in CRC cell lines, and its effects on proliferation, cell cycling, migration, invasion, cellular energy metabolism, apoptosis, chemotherapeutic drug sensitivity and cell phenotype‐related molecules were assessed. The growth of xenograft tumours in nude mice was also assessed. MiRNAs that potentially targeted SSRP1 were determined by bioinformatic analysis, Western blotting and luciferase reporter assays. We showed that SSRP1 mRNA levels were significantly increased in CRC tissue. We also confirmed that this upregulation was related to the terminal tumour stage in CRC patients, and high expression levels of SSRP1 predicted shorter disease‐free survival and faster relapse. We also found that SSRP1 modulated proliferation, metastasis, cellular energy metabolism and the epithelial‐mesenchymal transition in CRC. Furthermore, SSRP1 induced apoptosis and SSRP1 knockdown augmented the sensitivity of CRC cells to 5‐fluorouracil and cisplatin. Moreover, we explored the molecular mechanisms accounting for the dysregulation of SSRP1 in CRC and identified microRNA‐28‐5p (miR‐28‐5p) as a direct upstream regulator of SSRP1. We concluded that SSRP1 promotes CRC progression and is negatively regulated by miR‐28‐5p.

RETRACTED

## 1 INTRODUCTION

Colorectal cancer (CRC) is one of the most commonly diagnosed cancers and one of the major causes of cancer mortality worldwide.^1^ CRC is often diagnosed at an advanced stage, is accompanied by metastasis, which is negatively correlated with patient survival, and CRC remains incurable.^2^, ^3^, ^4^ Therefore, the discovery of new diagnostic and prognostic markers and a better understanding of the molecular mechanisms of colorectal tumorigenesis and metastasis are urgently needed.

Structure‐specific recognition protein 1 (SSRP1), which is a subunit of the histone chaperone facilitates chromatin transcription (FACT) complex, is involved in almost all chromatin‐related processes, including DNA replication, repair and transcription.^5^, ^6^, ^7^, ^8^, ^9^ SSRP1 is not widely expressed in most mature tissues and is detectable in only a very limited number of adult cells.^10^ SSRP1 is highly expressed in the early stages of embryonic development, and its expression is reduced gradually in the organs as birth nears and postnatal life begins, which suggests that SSRP1 plays a role in maintaining the undifferentiated cell state.^10^, ^11^, ^12^ Moreover, SSRP1 is up‐regulated in various tumours, such as breast cancer and ovarian cancer, and is associated with a worse prognosis.^13^, ^14^, ^15^ RNA interference (RNAi) knocks down SSRP1, inhibits tumour transformation and impairs tumour cell viability, but nontumour cells can tolerate this knockdown well.^16^ An inhibitor of SSRP1, CBL0137, causes cell death via blocking SSRP1‐dependent p53 activation as well as the downregulation of a subset of nuclear factor‐kappaB (NF‐κB)‐dependent genes; CBL0137 has been developed for human use and is currently being investigated in cancer clinical trials.^17^, ^18^ These results imply that SSRP1 is a potential target in cancer therapy. However, the function, mechanism and clinical value of SSRP1 in CRC remain obscure. In addition, although SSRP1 has been shown to induce many types of human cancers, previous studies have concentrated only on its role in stimulating proliferation by promoting cell cycle progression; its functions in metastasis and chemoresistance have rarely been investigated. Another problem to address is the mechanism underlying high SSRP1 expression in cancer tissue. MicroRNAs (miRNAs) are small noncoding RNA molecules that are highly conserved and can induce mRNA cleavage or repress translation by targeting the 3’UTR of corresponding mRNAs.^19^, ^20^, ^21^ Recently, an increasing number of studies have reported that miRNAs can regulate various cellular processes in cancer, such as proliferation, apoptosis, metastasis and chemoresistance.^20^ In this study, we have been suggested that the abnormal expression of SSRP1 in CRC is partly due to the upstream dysregulation of miRNAs.

RETRACTED

In this study, we provided the first data regarding the expression levels of SSRP1 and its clinical significance in human CRC. We found that SSRP1 is up‐regulated in CRC and significantly affects not only proliferation but also metastasis and chemosensitivity in CRC. We also showed the negative regulation of SSRP1 levels by microRNA‐28‐5p (miR‐28‐5p). In conclusion, we found that SSRP1 is an important oncogene in CRC, and the pathogenic up‐regulation of SSRP1 is partially attributed to the down‐regulation of miR‐28‐5p.

## 2 MATERIALS AND METHODS

### 2.1 Patients and immunohistochemistry

Colorectal cancer samples and paired nonneoplastic tissue were obtained from Renmin Hospital of Wuhan University. Immunohistochemical (IHC) staining of formalin‐fixed, paraffin‐embedded sections was performed using a streptavidin‐peroxidase IHC kit (Boster Biological Technology Co. Ltd., Wuhan, China) according to the manufacturer’s instructions. SSRP1 protein levels were assessed by two experienced pathologists. The mRNA expression profiles for GSE14333, GSE39582, GSE4107, GSE32323, GSE29623, GSE17536 and GSE35834 were downloaded from the GEO database (https://www.ncbi.nlm.nih.gov/gds).

### 2.2 Cell culture, small interfering RNAs and antibodies

HCT116, SW480, SW620, DLD‐1, LOVO and NCM460 cells were maintained in Roswell Park Memorial Institute 1640 medium (Invitrogen, CA, USA) supplemented with 10% foetal bovine serum (FBS) (GIBCO/BRL, MD, USA), 100 U/mL penicillin and 100 mg/mL streptomycin (Beyotime Biotechnology Co., Ltd, Shanghai, China). The cells were cultured at 37°C in 5% CO_2_. An siRNA targeting the SSRP1 transcript and a nonspecific control siRNA were purchased from Guangzhou RiboBio (Guangzhou RiboBio Co., Ltd, Guangzhou, China). The target sequences for the SSRP1 transcript were as follows: siRNA‐1: GCCATGTCTACAAGTATGA; siRNA‐2: GCCCAGAATGTGTTGTCAA; and siRNA‐3: GCATTACCTGTTCCTACAA. The specific siRNA or negative control was transfected into CRC cells with Lipofectamine 2000 transfection reagent (Invitrogen) in accordance with the manufacturer's instructions. Antibodies against SSRP1 (15696‐1‐AP), E‐cadherin (20874‐1‐AP), N‐cadherin (22018‐1‐AP), ZO‐1 (21773‐1‐AP), ZEB1 (21544‐1‐AP), ZEB2 (14026‐1‐AP), SNAI (13099‐1‐AP), SLUG (12129‐1‐AP), Twist (18125‐1‐AP), Bax (50599‐2‐Ig), Bcl‐2 (12789‐1‐AP), VEGF (19003‐1‐AP), cyclin D1 (0186‐1‐Ig), and MMP9 (10375‐2‐AP) were purchased from Proteintech Group; antibodies against p53 (#2527s) and Flag (#2368s) were purchased from Cell Signalling Technology (MA, USA); antibodies against 14‐3‐3 (sc‐69720) and GAPDH (sc‐47724) were purchased from Santa Cruz Biotechnology, Inc (CA, USA); antibodies against p21 (#3733‐1) and p27 (#2747‐1) were purchased from Epitomics, Inc (CA, USA).

RETRACTED

### 2.3 Western blotting

Colorectal cancer proteins were separated by SDS polyacrylamide gel electrophoresis. Proteins were transferred onto a polyvinylidene fluoride membrane and incubated for 60 minutes in TBST (0.05% Tween‐20 in phosphate‐buffered saline) with 5% dried skim milk at room temperature. Immunoblot analysis was performed using the appropriate primary antibody at 4°C for 12 hours. After being washed three times, the membranes were incubated with a horseradish peroxidase conjugated secondary antibody for 60 minutes. Immunoreactive bands were visualized with an enhanced chemiluminescent detection kit (Beyotime Biotechnology Co., Ltd).

### 2.4 Quantitative real‐time PCR

Total RNA was isolated from cell lines and human tissues using an RNA isolation kit (Takara Biomedical Technology (Beijing) Co., Ltd.). We used M‐MLV reverse transcriptase to synthesize cDNA. A SYBR Green reaction system (Takara Biomedical Technology (Beijing) Co., Ltd.) was used to amplify the cDNA. The differences in SSRP1 RNA expression were normalized to the corresponding GAPDH RNA signals. The PCR primers used were as follows: SSRP1: sense: 5‐GTGTTGTCAAAGGCGGATGT‐3, antisense: 5‐ACAAAGAACATCTGGCGCTG‐3; and GAPDH: sense: 5‐GTGGACATCCGCAAAGAC‐3, antisense: 5‐AAAGGGTGTAACGCAACTA‐3.

### 2.5 Cell viability assays with Cell Counting Kit‐8 and xCELLigence real‐time cell analysis system

Cells proliferation assays were performed with Cell Counting Kit‐8 reagent (Dojindo, Japan) according to the manufacturer’s instructions. For CCK‐8 proliferation analysis, the cells were seeded in 96‐well plates, and the total cell number was determined at the indicated time points. Additionally, the cells were seeded in 16‐well E‐plates for xCELLigence assays. The analyser was placed in a standard cell incubator and the cells were cultured for 48 hours to dynamically monitor cell proliferation in real time.

### 2.6 Metabolic analyses

The oxygen consumption rate (OCR) and extracellular acidification rate (ECAR) were measured with an XF Extracellular Flux Analyser (Seahorse Bioscience). We used a protocol previously described.^22^ The data were analysed using Seahorse XF software. OCR and ECAR measurements were normalized to either the final cell number or the protein concentration.

RETRACTED

### 2.7 Cell cycle analysis

One million cells were used for the cell cycle analyses. The cells were fixed in cold methanol for at least 2 hours and then incubated with a propidium iodide (PI)/RNase A solution. The cell cycle distribution was assessed with a FACSCalibur system (Becton‐Dickinson, NJ, USA). Modfit 2.0 software was used to detect the percentage of cells in different phases.

### 2.8 Apoptosis analysis

Apoptotic cells were detected by Annexin V/PI staining (Life Technologies, CA, USA) and measured by flow cytometry. The experiments were performed in triplicate. The results represent the means ± SD. FlowJo7.6.1 software was used to analyse the ratio of apoptotic cells.

### 2.9 Migration and invasion assays

In vitro tumour cell motility was measured using transwell migration chambers (Corning, NY, USA) and invasion chambers (BD Biosciences, CA, USA). In brief, 2 × 10^5^ cells with/without siRNA in 2% FBS‐supplemented medium were plated in the upper chamber, and media supplemented with 10% FBS was added to the bottom chamber for 48 hours. Subsequently, the cells that migrated/invaded to the bottom of the upper membrane were stained with 0.1% crystal violet dye. The number of cells was determined from five random fields viewed under a microscope.

### 2.10 In vivo tumorigenicity assay

Male BALB/C nude mice that were 5 weeks old and weighed 20‐22 g were provided by the Beijing Vital River Laboratory Animal Technology Co., Ltd. The mice were randomly assigned to the experimental or control group (six mice per group). A total of 4 × 10^6^ HCT116 cells infected with the GV358‐SSRP1 virus were injected on the mice. GV358‐vector infected cells were used in the control group. The tumours were measured every 3 days, and the tumour volumes were calculated using the formula: length (mm) × width (mm) × height (mm) × 0.5.

### 2.11 Chemotherapeutic drug sensitivity analysis by Cell Counting Kit‐8 assay

Colorectal cancer cells were treated with various concentrations of the chemotherapeutics 5‐fluorouracil and cisplatin for 72 hours. Cell viability was determined using a Cell Counting Kit‐8 assay (Dojindo, Japan) according to the manufacturer’s instructions. The sensitivity of the CRC cells to the chemotherapeutic drugs was assessed by the IC_50_ value measurement.

### 2.12 Luciferase assay

We obtained pMIR‐REPORT luciferase plasmids (Obio Technology (Shanghai) Corp., Ltd., China) that contain the 3’UTR region of the human SSRP1 gene and a mutant 3UTR region of the human SSRP1 gene. The cells in 12‐well plates were cotransfected with 200 ng of the pMIR‐REPORT plasmids and 100 nmol/L miR‐28‐5p (or control miRNA). Lysates were obtained 48 hours after transfection. Firefly and Renilla luciferase activities were measured with a dual‐luciferase reporter system (Promega) according to the manufacturer’s instructions.

RETRACTED

### 2.13 Statistical analysis

Each experiment was performed at least three times. Survival analyses were statistically analysed by the log‐rank test. The unpaired Student’s *t* test and one‐way ANOVA were used to analyse the differences between two variables and multiple variables, respectively. A significant difference was defined as *P* < 0.05.

## 3 RESULTS

### 3.1 SSRP1 expression is up‐regulated in CRC

We first analysed SSRP1 mRNA expression in CRC patients from two independent GEO datasets, GSE32323 and GSE4107. The two datasets included paired CRC tumour and adjacent noncancerous tissue mRNA information. As shown in Figure 1A, SSRP1 mRNA levels were significantly higher in human colorectal tumour tissue than those in adjacent normal colorectal tissue.

**Figure 1:** SSRP1 expression is upregulated in CRC. A, SSRP1 expression levels in CRC tissue and normal tissue in two independent cohorts (GSE32323 and GSE4107). B, SSRP1 mRNA expression levels in 10 paired tissue tumour samples and normal tissue samples. C, SSRP1 protein expression levels in five CRC cell lines and the normal colon NCM460 cell line. D and E, Representative photographs of IHC staining for SSRP1 in normal and CRC tissue. F, SSRP1 expression was up‐regulated in 85% of CRC patients according to IHC. *P < 0.05, **P < 0.01, and ***P < 0.001. IHC: immunohistochemical staining

To verify the microarray analysis results, we performed qRT‐PCR experiments on human colorectal adenocarcinoma specimens and their paired normal tissues. Compared with their respective matched normal tissue, nine of the ten tumour samples showed increased SSRP1 mRNA levels (Figure 1B). Moreover, SSRP1 expression was determined by Western blot for several CRC cell lines, including DLD‐1, LOVO, SW620, SW480 and HCT116 cells, as well as the normal colon cell line NCM460. According to the results, observably higher expression levels of SSRP1 were found in most CRC cells compared to those of NCM460 cells (Figure 1C). To further investigate the connection between SSRP1 and CRC progression, we also measured the expression levels of SSRP1 in 80 human CRC tissue samples (Table S1; 60 cases of colon cancer and 20 cases of rectal carcinoma) and their paired normal tissue. SSRP1 was located in the cytoplasm and nucleus (Figure 1D,E), which was in accordance with the results of previous reports.^17^, ^23^ As shown, SSRP1 was up‐regulated in the majority (85%, 68/80) of the CRC specimens (Figure 1F). In conclusion, these data clearly indicated that SSRP1 was up‐regulated in CRC at both the mRNA and protein levels, which hinted at the importance of SSRP1 in the pathogenesis of CRC.

RETRACTED

### 3.2 SSRP1 expression levels are correlated with disease progression and shortened patient survival

To confirm the correlation between SSRP1 expression levels and clinicopathological factors in CRC, the clinical information for GSE14333 was downloaded and statistically analysed. The pooled samples in the dataset were then divided into two groups based on the SSRP1 expression level in the tumour tissue, and the chi‐squared test was applied. As shown in Table 1, higher SSRP1 expression level was closely related to the Dukes stage (*P* = 0.003). The results suggested that high SSRP1 expression was associated with rapid carcinoma spread. Importantly, the results showed that CRC patients with tumours with high SSRP1 expression levels had markedly shorter DFS and RFS than those with tumours with low SSRP1 expression (Figure S1A,B) (*P* = 0.0025 and *P* = 0.019, respectively). These findings strongly suggest that SSRP1 may be a new prognostic factor for CRC.

**Table 1:** Correlations between the SSRP1 expression and the clinicopathologic features of the colorectal carcinoma cohort (GSE14333)

Characteristics	No. of patient	SSRP1 expression		Chi‐squared value	*P* value
		High	Low		
Age					
>60	200	101	99	−0.253	0.800
≤60	90	44	46		
Gender					
Male	164	75	89	−1.656	0.098
Female	126	70	56		
Location					
L‐colon	138	68	70	0.663	0.718
R‐colon	111	55	56		
Rectum	39	22	17		
Ducks stage					
A	44	16	28	13.919	0.003
B	94	38	56		
C	91	51	40		
D	61	40	21		

Data are presented as number.

L‐colon: Left half colon; R‐colon: Right half colon.

### 3.3 SSRP1 modulates CRC cell proliferation in vitro and in vivo

To verify the biological role of SSRP1 in CRC cell proliferation, we depleted SSRP1 in HCT116 and SW480 cells using three siRNAs. After transfecting the three siRNAs into CRC cells, we used Western blot analysis to measure the SSRP1 protein levels. Figure S2A shows that all the targeted siRNAs could knock down SSRP1 effectively in the two cell lines compared with the control siRNA; siRNA‐2 was the most effective; thus, this siRNA was chosen to do the following verification. SSRP1 was stably overexpressed by the lentivirus‐mediated delivery of the pLV‐SSRP1 plasmid in the HCT116 cell line, which has a relatively lower level of SSRP1 expression compared to the expression in the other CRC cell lines. The expression of SSRP1 in the cells was verified by fluorescence microscopy, Western blotting and qRT‐PCR (Figure S2B‐D). As expected, cell proliferation was suppressed significantly by SSRP1 siRNA interference in SW480 (Figure S3A) and HCT116 cells (Figure 2A), and it was enhanced by the overexpression of SSRP1 in HCT116 cells (Figure 2A).

RETRACTED

**Figure 2:** SSRP1 modulates CRC cell proliferation and the cell cycle in HCT116 cells. A, SSRP1 knockdown or overexpression reduced or accelerated the proliferation rate of cells, respectively. B, Representative data show that the overexpression of SSRP1 significantly promoted tumour growth in a nude mouse xenograft model (n = 6). C, Tumours were dissected, and tumours from the two groups are shown. D, The effects of SSRP1 knockdown on the cell cycle were determined. The percentages of cells in the G1, S and G2/M phases of the cell cycle are presented. The bars represent the mean values of six independent tests (mean ± SD). E, The effects of SSRP1 overexpression on the cell cycle were determined. F, Cell cycle‐related molecules were screened by Western blot analysis, and SSRP1 expression levels altered the expression of cell‐cycle‐related proteins in HCT116 cells. *P < 0.05, and **P < 0.01. p21: cyclin‐dependent kinase inhibitor 1A; p27: Cyclin‐dependent kinase inhibitor 1B; 14‐3‐3: YWHAS, epithelial cell marker protein 1

To verify the effect of SSRP1 on CRC progression in vivo, we performed xenograft tumour assays using HCT116 cells stably transfected with SSRP1‐overexpression lentiviruses or control lentiviruses. We found that the lentiviral expression of SSRP1 resulted in accelerated xenograft tumour growth (Figure 2B,C). These data collectively demonstrate that SSRP1 expression is closely related to the proliferation of CRC cells.

Cell proliferation depends largely on cell cycle progression. Hence, the impact of SSRP1 knockdown on the cell cycle process was also assessed by flow cytometry. After treatment with si‐SSRP1 or control siRNA for 48 hours, the cells were collected and stained with PI. SSRP1 knockdown resulted in an obvious accumulation of cells in the G0/G1 phase and a considerable decrease in the proportion of cells in the S/G2/M phases in HCT116 (Figure 2D) and SW480 cells (Figure S3B); in contrast, the overexpression of SSRP1 promoted cell cycle progression in HCT116 cells (Figure 2E). These data suggest that SSRP1 modulates the cell cycle. We proceeded to determine the expression levels of p53, which is a key cell cycle regulator.^24^ As shown in Figure 2F, we determined p53 expression levels after SSRP1 knockdown and found that SSRP1 knockdown led to an increase in p53 protein levels. We further examined several p53 downstream cell‐cycle‐related molecules and found that p21 and p27 were up‐regulated following SSRP1 knockdown in HCT116 cells. The expression levels of cyclin D1 and 14‐3‐3, which is a cyclin negatively regulated by p21, were reduced in SSRP1 knockdown cells. Moreover, the overexpression of SSRP1 had the opposite effect.

RETRACTED

These results showed SSRP1 regulates p53 and its related downstream molecules. The regulation of the p53 pathway by SSRP1 might be the underlying mechanism of SSRP1‐mediated cell cycle progression in CRC cells.

### 3.4 SSRP1 modulates cell phenotypes and associated molecules in CRC

The role of SSRP1 has not been well characterized in cancer metastasis. We determined whether SSRP1 is a key molecule that has an impact on cell migration and invasion by transwell assay. As shown, knocking down SSRP1 inhibited the migration and invasion rates of SW480 and HCT116 cells (Figure 3A,B); in contrast, the forced expression of SSRP1 had the opposite effect on HCT116 cells (Figure 3C). These results demonstrated that the expression level of SSRP1 is positively related to cell migration and invasion. It is well known that VEGF and MMP9 are critical proteins for cancer cell invasion and metastasis and that the autocrine secretion of these cytokines by cancer cells critically influences cancer cell behaviours such as invasion.^25^ When SSRP1 was knocked down in HCT116 cells, MMP9 and VEGF were down‐regulated (Figure 3D), and the opposite regulation was seen in SSRP1‐overexpressing cells.

**Figure 3:** SSRP1 modulates cell motility and phenotype‐related molecules in CRC. A, Cell migration was assessed by transwell migration assay in SSRP1 knockdown cells. B, Cell invasion was assessed by transwell invasion assay in SSRP1 knockdown cells. C and D, Cell migration and invasion were assessed by transwell assay in SSRP1 overexpressing cells. E, Phenotype‐related molecules were screened by Western blot analysis

The epithelial‐mesenchymal transition (EMT) plays an important role in cancer progression and metastasis.^26^ Given that SSRP1 promotes the migration and invasion of CRC cell lines, we next tested whether SSRP1 affects the EMT process in CRC. Consistent with our hypothesis, the protein expression levels of the epithelial markers ZO‐1 and E‐cadherin were obviously decreased in stable SSRP1‐overexpressing HCT116 cells; in contrast, the expression levels of the mesenchymal markers Snail, Slug, ZEB1, ZEB2, N‐cadherin and Twist were dramatically increased (Figure 3D). Corresponding results were obtained with SSRP1‐knockdown HCT116 cells (Figure 3D). Collectively, our results show that SSRP1 contributes to the promotion of EMT in CRC cells, which at least partly explains why SSRP1 overexpression promotes metastasis and invasion in CRC cells.

Many oncogenes or tumour suppressor genes are deregulated during tumorigenesis, which leads to the abnormal cellular bioenergetics that give cancer cells a growth advantage. Increases in glycolysis and mitochondrial biogenesis are the most prominent metabolic alterations in cancer.^22^ The ECAR is an indicator of glycolysis, and the OCR is an indicator of mitochondrial respiration. Hence, the impacts of SSRP1 on ECAR and OCR were also assessed. SSRP1‐overexpressing CRC cells showed a higher rate of glycolysis and a higher mitochondrial respiratory ratio than the mock‐treated and control cells according to the ECAR and OCR, while SSRP1 knockdown had the inverse effect (Figure S4A,B).

RETRACTED

These data show that SSRP1 promotes malignant progression by promoting CRC cell motility and increasing glycolysis and aerobic oxidation.

### 3.5 SSRP1 modulates the sensitivity of CRC cells to chemotherapeutic drugs

After exploring the function of SSRP1 in CRC cell growth and metastasis, we attempted to determine whether SSRP1 could be used for clinical CRC treatment. Chemotherapy is an important strategy for the treatment of CRC. However, primary and secondary drug resistance is a major challenge in basic and clinical research, which greatly reduces the antitumour efficacy of therapy in many cases.^27^ We first determined the effects of SSRP1 on apoptosis with or without cisplatin treatment. Under these two conditions, SSRP1 knockdown markedly increased the number of apoptotic SW480 (Figure 4A) and HCT116 (Figure 4B) cells. The negative effect of SSRP1 on apoptosis in CRC cells prompted us to hypothesize that SSRP1 may also contribute to the drug resistance of CRC cells. Therefore, we determined the chemosensitivity of the two cell lines to the two most frequently used chemotherapy drugs, cisplatin and 5‐fluorouracil, in the SSRP1 knockdown and control groups. The results showed that the IC_50_ values of both chemotherapy drugs decreased significantly in the two CRC cell line groups with SSRP1 knockdown (Figure 4C). Together, these data indicated that SSRP1 beneficially reduced the sensitivity of CRC cells to chemotherapeutic drugs.

**Figure 4:** SSRP1 modulates the sensitivity of CRC cells to chemotherapeutic drugs. A and B, SSRP1 knockdown promotes cell apoptosis. C, siRNA‐mediated SSRP1 knockdown increases the sensitivity of CRC cells to chemotherapeutics

Cell apoptosis is closely associated with the regulation of apoptosis‐related genes, including Bcl‐2.^28^ To determine the mechanisms by which SSRP1 regulates apoptosis and chemoresistance, the expression of apoptosis‐related proteins in HCT116 cells with SSRP1 knockdown or stable overexpression was examined by Western blotting. As shown in Figure S5, si‐SSRP1 transfection induced the expression of Bax (a molecule indicating a proapoptotic phenotype) and decreased the expression of Bcl‐2 (a molecule indicating an antiapoptotic phenotype). In contrast, SSRP1 overexpression had inverse effects on HCT116 cells.

RETRACTED

Collectively, our results show that SSRP1 promotes the sensitivity of CRC cells to chemotherapeutic drugs by promoting cell apoptosis.

### 3.6 Identification of SSRP1 as a new target for miR‐28‐5p

MiRNAs play an important role in gene expression regulation. It would be interesting to confirm whether a specific miRNA could regulate SSRP1 expression in CRC. Potential miRNAs that target the 3UTR of SSRP1 were predicted, and their target sites were analysed by TargetScan, miRanda and miRwalk. To reduce false positives, candidates were considered only if they were predicted by all three methods. One candidate identified by this approach was miR‐28‐5p, which has one site complementary to the 3UTR of SSRP1 (Figure 5A). It has been confirmed that miR‐28‐5p is down‐regulated in CRC; we also verified this by analysing the GEO datasets (Figure 5B). Furthermore, the overexpression of miR‐28‐5p inhibited CRC cell proliferation, migration, and invasion.^29^ Importantly, Kaplan‐Meier survival analysis suggested that CRC patients with tumours with low miR‐28‐5p expression levels had observably shorter DFS times than those with tumours with high miR‐28‐5p expression (Figure 5C) (*P* = 0.015). Therefore, we proposed that the overexpression of SSRP1 was partly attributed to the down‐regulation of miR‐28‐5p. After transfection with miR‐28‐5p, we observed that SSRP1 protein levels decreased in SW480 and HCT116 cells (Figure 5D). We found that miR‐28‐5p could suppress the reporter gene activity of SSRP1 in HEK293T cells; in addition, the suppression was weaker when the mutation plasmid (MT plasmid) was used (Figure 5E). These data indicated that SSRP1 was a direct target of miR‐28‐5p. A negative correlation was also observed between miR‐28‐5p and SSRP1 expression levels in CRC samples (Figure 5F; *P* < 0.0001, *R* = −0.731). These data support the idea that SSRP1 expression is negatively regulated by miR‐28‐5p in CRC.

**Figure 5:** Identification of SSRP1 as a novel target for miR‐28‐5p. A, The miR‐28‐5p target sites in the 3’UTR of SSRP1 are shown as a schematic representation. B, miR‐28‐5p expression levels in CRC tissue and adjacent/normal tissue from the mRNA microarray data obtained from GSE35834. C, Low miR‐28‐5p levels were associated with decreased disease‐free survival in CRC patients in the GSE29623 dataset. D, Western blotting showed the expression of SSRP1 protein in SW480 and HCT116 cells transfected with miR‐28‐5p. E, Wild‐type or mutant 3’UTR constructs of SSRP1 were cloned into a pMIR‐REPORT luciferase vector and cotransfected with miR‐28‐5p mimics into HEK293 cells. Renilla luciferase activity was normalized to firefly luciferase activities. All assays were performed in triplicate and repeated at least three times. F, An inverse correlation was found between miR‐28‐5p expression and SSRP1 expression in CRC samples (GSE29623 dataset) (Spearman’s correlation, *P* < 0.0001, *R* = −0.731). The data are expressed as the mean ± SD of three independent experiments; **P < 0.01, and ***P < 0.001

RETRACTED

## 4 DISCUSSION

Our study shows that SSRP1 promotes CRC progression, which agrees with previous studies in other types of cancers, such as nonsmall cell lung cancer,^30^ breast cancer^13^, ^31^ and hepatic carcinoma (HCC).^23^ Significantly shortened survival is observed in patients with high SSRP1 expression compared with patients with low SSRP1 expression. Our data suggest that SSRP1 knockdown inhibited the cell cycle and promoted apoptosis in CRC cells in vitro, which may result in slower cancer cell proliferation in vivo. However, the underlying mechanism is still unclear, and several possible explanations are put forward here.

First, a hallmark of cancer cells is that they maintain proliferative ability, which can be achieved by inactivating tumour‐suppressor genes and dysregulating tumour‐associated transcription factors. P53 is a widely known tumour suppressor.^32^ The deregulation of the transcription factor NF‐κB is a common event in many types of cancers that are susceptible to tumour initiation and progression via the expression of proproliferative/antiapoptotic genes.^33^ It has been reported that the NF‐κB and p53 pathways can be modified by the FACT complex.^13^, ^30^ Curaxins can effectively bind the heterodimeric protein complex FACT, and the sequestration of FACT leads to the regulation of various pathways (p53 activation and NF‐κB inhibition), resulting in tumour cell death without DNA damage.^17^, ^18^, ^34^ Hence, the activation of the NF‐κB pathway and the suppression of the p53 pathway could be considered a mechanism underlying SSRP1 function in CRC tumorigenesis.

P53 expression is associated with cell cycle arrest.^24^ Moreover, cell cycle proteins, such as p21 and p27, are the signalling factors downstream of p53, which can be regulated by p53. In addition, the expression levels of cyclin D1 and 14‐3‐3 can be negatively regulated by p21. The p27 amino‐terminal region has 44% similarity with p21, which prevents cells moving from the G0/G1 to S phase transition.^35^ In this paper, we measured the expression of p53 and its downstream signalling molecules p21, p27, cyclin D1 and 14‐3‐3 after inhibiting or overexpressing SSRP1 in cells. We found that the siRNA‐induced knockdown of SSRP1 significantly inhibited cell cycle progression from G0/G1 phase to S phase in CRC cells, resulting in G1 cell cycle arrest due to the reduction in cyclin D1 and 14‐3‐3 expression and the increase in p53, p21 and p27 expression. Moreover, the overexpression of SSRP1 had the opposite effect. The regulation of the p53 pathway by SSRP1 might be the underlying mechanism of SSRP1‐mediated cell cycle arrest in CRC cells. The results show that SSRP1 regulates p53 and its related downstream molecules, and this regulation may enhance the malignant biological behaviour of SSRP1‐overexpressing CRC cells.

RETRACTED

In addition, cancer cells maintain proliferative signalling, which is accompanied by enhanced DNA replication.^36^ SSRP1 is a key regulator maintaining DNA replication in the normal cell process.^37^ SSRP1 knockdown inhibited cell growth due to the inhibition of duplication fork progression.^38^ Furthermore, it has been reported that SSRP1 is involved in canonical Wnt/β‐catenin‐mediated signalling pathways.^11^ The activation of the Wnt/β‐catenin signalling pathway also plays a key role in the formation of CRC; mutations in the negative regulatory components of APC occur in more than 90% of colorectal tumours.^39^ We have been suggested that the high expression levels of SSRP1 regulate the Wnt/β‐catenin pathways in CRC. In the present study, when SSRP1 was knocked down or overexpressed, the signalling molecules downstream of the Wnt/β‐catenin pathway and those associated with EMT changed significantly. Therefore, we speculated that SSRP1 may promote the malignant biological behaviour of CRC cells by promoting EMT via the Wnt/β‐catenin pathway. Lastly, the expression levels of MYC and FACT are obviously higher in malignant tissue than those in normal tissue.^10^, ^15^, ^40^ The MYC oncogene is believed to be involved in more than half of human tumours.^3^ There is an interaction between MYC and FACT that causes MYC to directly drive the transcription of SUPT16H and SSRP1, and FACT then positively regulates MYC expression and protein stability in turn.^41^ Animal models with conditional gene knockout of SSRP1 or Spt16 have revealed the specific functions of FACT in neuroblastoma development and, by association, in MYC‐driven tumorigenesis.^41^ These reports suggest several possible mechanisms by which SSRP1 may regulate malignant cell progression in CRC.

In our work, we confirmed that SSRP1 modulates not only proliferation but also motility, migration, invasion and chemosensitivity. In CRC, metastasis is the most fatal event during disease progression; it accounts for approximately 90% of patient deaths.^42^ Metastasis is inversely related to the survival of the patient and critically limits successful therapy.^43^ Metastasis formation is a major obstacle in CRC therapy. Therefore, the identification of high‐risk patients with metastasis formation and the early diagnosis and molecular characterization of primary tumours are vital steps to determine prognostic and therapeutic markers.^44^ Our results suggest that SSRP1 is an important target for impeding metastasis in CRC. Chemotherapy is one of the most effective methods of treatment. However, aberrant cell signalling activation and exceptional changes in some oncogenes often lead to uncontrolled drug resistance, recurrence and metastasis.^45^ During carcinogenesis, EMT results in a loss of polarity in epithelial cells and the transformation of epithelial cells into mesenchymal cells. As a result of EMT, tumour cells show characteristics of cancer stem cells with superior tumorigenic effects and develop more powerful drug resistance to promote tumour relapse and metastasis.^46^ Increasing evidence shows the potential role of EMT in the development of drug resistance. Patients with EMT often have a poor quality of life compared to those who do not develop EMT.^47^ In our study, SSRP1 was identified to participate in the regulation of EMT in CRC, so SSRP1 may be a vital target for reversing drug resistant properties in CRC. We propose that the quantification of SSRP1 in colon biopsies could be used in combination with pathologic examinations to forecast the biological behaviours of CRC. The molecular pathological diagnosis will be helpful for optimizing individual treatments.

RETRACTED

MiRNAs play an important role in transcriptional regulation by acting on the 3'UTR of target genes that participate in various biological processes. MiRNAs can affect tumour growth positively or negatively by controlling the expression of oncogenes and tumour‐suppressor genes. The down‐regulation of miR‐28‐5p has been reported in multiple cancers, such as renal cell carcinoma,^48^ CRC^49^, ^50^ and HCC.^51^ Increasing evidence indicates that miR‐28‐5p negatively regulates a number of well‐characterized oncogenic proteins, such as CCND1, HOXB3,^29^ IL‐34, FAK, ERK1/2^51^ and insulin‐like growth factor 1.^52^ In this study, miR‐28‐5p expression was down‐regulated in CRC samples compared with that in normal colon samples, and the down‐regulation of miR‐28‐5p forecasted a poor prognosis for CRC patients, suggesting that this miRNA plays a tumour‐suppressive role. Most cells in human tissue do not express SSRP1 at the protein level, but SSRP1 is expressed at high levels in undifferentiated or cancerous tissues; however, the mechanisms of SSRP1 up‐regulation have not yet been determined in cancer. Our work showed that SSRP1 is a new target of miR‐28‐5p and that there is a negative relationship between miR‐28‐5p and SSRP1 expression. Taken together, these results reveal a novel regulatory pathway employing miR‐28‐5p and SSRP1 to fine‐tune the balance of CRC.

RETRACTED

In summary, our study has shown the biological and clinical significance of SSRP1 in CRC. Our study demonstrated that SSRP1 expression is observably up‐regulated in CRC tissue and is correlated with the Dukes stage of the tumour. SSRP1 is a newly identified target of miR‐28‐5p; this finding partially explains the abnormally high expression of SSRP1 in cancers. Our evidence provides novel clues that may aid CRC diagnosis and treatment in the future. However, it will be necessary to further explore the molecular mechanisms of SSRP1 in promoting proliferation, metastasis and drug resistance in depth.

## ETHICAL APPROVAL

The inclusion of human samples was approved by the Ethics Review Board of the Second People’s Hospital of Guangdong Province (approval no. 2015‐KYLL‐023). All animal experiments were approved by the Ethics Review Board of the Second People's Hospital of Guangdong Province (approval no. 2015‐KYLL‐063).

## CONFLICT OF INTEREST

The authors confirm that there are no conflicts of interests.

## AUTHOR CONTRIBUTION

QSD, GAX, HGY, XL conceived and designed the experiments and coordinated; GAX, HGY, QSD, QG provided the funds and materials; WW, KH(e), QG, KH(uang), JDC, MJZ, DMY, LW, YCD performed the experiments and interpretation; WW conducted the bioinformatics and statistical analysis; WW, JDC, MJZ, HGY and QSD wrote this manuscript. All the authors have read and approved the final edition of this manuscript.
